# Design of Bionic Buffering and Vibration Reduction Foot for Legged Robots

**DOI:** 10.1155/2021/5510993

**Published:** 2021-06-09

**Authors:** Qian Cong, Xiaojie Shi, Ju Wang, Yu Xiong, Bo Su, Lei Jiang, Ming Li, Weijun Tian

**Affiliations:** ^1^Key Laboratory of Bionic Engineering, Ministry of Education, China, Jilin University, Changchun 130022, China; ^2^State Key Laboratory of Automotive Simulation and Control, Jilin University, Changchun 130022, China; ^3^North-Vehicle Research, Fengtai District, Beijing 100072, China; ^4^Sany Group Co. Ltd., Changsha, Hunan, China

## Abstract

When legged robots walk on rugged roads, they would suffer from strong impact from the ground. The impact would cause the legged robots to vibrate, which would affect their normal operation. Therefore, it is necessary to take measures to absorb impact energy and reduce vibration. As an important part of a goat's foot, the hoof capsule can effectively buffer the impact from the ground in the goat's running and jumping. The structure of the hoof capsules and its principle of buffering and vibration reduction were studied. Inspired by the unique shape and internal structure of the hoof capsules, a bionic foot was designed. Experimental results displayed that the bionic foot could effectively use friction to consume impact energy and ensured the stability of legged robot walking. In addition, the bionic foot had a lower natural vibration frequency, which was beneficial to a wide range of vibration reduction. This work brings a new solution to the legged robot to deal with the ground impact, which helps it adapt to a variety of complex terrain.

## 1. Introduction

Mobile robots had received much attention in the past few years because they could play an important role in rescue operation, space exploration, and so on [1–4]. Though wheeled and tracked robots could run well in flat terrain, most of them could not adapt to working in complex and cluttered terrain. The legged robots have more potential to walking on almost all the earth surfaces in different terrains, just like humans and animals [5–7]. When legged robots walk or jump, they need to face many problems such as contact impact with friction from the ground. It is a complex work to characterize the contact impact because there are a lot of factors that need to be taken into account such as material properties and contacting surfaces [8, 9]. Scientists proposed many different types of contact force models. Corral et al. reported a general approach for the dynamic modeling and analysis of a passive biped walking robot, with a particular focus on the feet-ground contact interaction. They evaluated different kinds of contact forces in robot walking by several force models. The experiment result displayed that a dissipative nonlinear Flores contact force model worked best [10].

These feet-ground contact impacts would cause the legged robot to vibrate, which would affect their walking stability, control precision, and service life [11–13]. Researchers and engineers proposed a variety of methods to absorb impact energy and reduce vibration such as flexible feet [14]. Li et al. designed a flexible foot for the humanoid robot, which included a landing impact absorption mechanism and a foot attitude estimation system [15]. The rubber bushes and pads were utilized for absorbing impacts. Hashimoto et al. reported a foot cushion device for the WL-16 robot. It adopted a cam self-locking mechanism, which could be actively adjusted and controlled according to the force feedback of the contact position. This mechanism successfully helped the robot to reduce the vibration [16]. Zhu designed a novel kind of flexible robotic foot. The bottom of the robot foot was integrated with a spring-damping system, which was composed of spring, damper, rubber pad, etc. The system not only had a good vibration reduction effect but also had an excellent service life [17]. Kim and Yoon proposed an intelligent robot foot which could greatly reduce the vibration caused by uneven ground. The foot intelligently adjusted its position according to the force and moment of the sole [18]. Although the traditional buffering and vibration reduction mechanism for legged robots has made good progress, there are still some problems to solve such as high cost and complex manufacturing. By finding out excellent cushioning and vibration reduction features of biological structures, scientists and engineers have designed and manufactured lots of bionic vibration reduction devices [19]. Chang et al. proposed a bionic robot foot based on the bone structure of the German shepherd dog. It could transform the rigid contact between the robot and the ground into flexible contact and reduce the vibration caused by the impact of the ground [20]. Jiang et al. designed a bionic multijoint vibration control platform based on the human legs. The platform achieved vibration reduction by the knee joint mechanism composed of rods and springs. The experimental results displayed that it had excellent nonlinear vibration damping effects in the low-frequency range [21].

In the last million years, quadrupeds have evolved a lot of unique biological structures, which help them to adapt to various environments and terrains [22]. As a typical quadruped, goats have an excellent ability to move, jump, and run on unstructured terrain [23, 24]. As an important part of goats that directly contacts the ground, the hoof capsule could withstand a great external impact instantly, absorb the impact, and effectively reduce the vibration brought by the impact [25–27] The hoof capsule was dissected, and its internal structure was studied. Based on the above works, a bionic buffering and vibration reduction foot was designed.

## 2. Bionic Foot Based on the Hoof Capsules of Goats

### 2.1. Treatment of Biomaterials

Adult and healthy white goats without limitation to gender (40 ± 0.5 kg) were bought from an abattoir of Changchun City. Their hoof capsules were cut off and made into samples. Firstly, the samples were washed with ultrapure water to remove dust. They were then washed with anhydrous ethanol and acetone to remove grease and other contaminants. The above steps were repeated three times. After that, the samples were put in anhydrous ethanol and sonicated for 20 min and then placed in a drying cabinet for 24 h. The hoof capsules finally were placed in vacuum film deposition equipment for gold spraying for 30 s, followed by observation under an EVO 18 scanning electron microscope (SEM, Carl Zeiss Microscopy GmbH, Jena, Germany).

### 2.2. Design of the Bionic Foot

As shown in Figure 1, the hoof capsules consisted of a hard nail and soft toe pillow, presenting an inverted V shape. This shape could help goats acquire a bigger contact area and friction [23, 28]. The combination of nails and toe pillows allowed the goat to adapt to hard rock surfaces and soft soil surfaces. When goats walk on hard ground like rocks or cliffs, the sunken soft toe pillow fitted with the hard ground to obtain a large contact area, further increasing friction and reducing impact pressure. When they move on soft ground such as muddy roads and sand, the hard nails would insert into them. Goats also get a larger contact area and friction, which helps them use friction to consume impact energy.

As an important part of the bionic foot, the robot foot sole needs to help the robot obtain greater friction force and contact area to ensure the stability of walking. Therefore, the touch curve of the hoof capsules was used to design the sole of the bionic foot. To obtain the contact curve, the hoof capsule coated with ink on the bottom was pressed firmly at a suitable position in the grid paper to obtain an imprint. The imprint was then scanned to obtain the contact contour (Figure 2(a)). The spline curve was used to fit the hoof capsules' contact contour. According to the feature that the nail was higher than the toe pillow, the bionic sole with protrusion was designed (Figure 2(b)). The shape of the protrusion was derived from the unilateral spline curve of the hoof capsules' contact contour. The design of the bionic sole could ensure that the robot can obtain a large contact area and better consume the impact energy from the ground through friction.

The SEM pictures of hoof capsules are displayed in Figure 3. The hoof capsule was composed of two layers of tissue. There were a lot of cornified tissues on the bottom of the hoof capsules, showing a layered shape. At the top of the hoof capsules, there was a layer of inclined holes with hexagonal distribution, which were round or oval. The distance between two adjacent holes was 140 *μ*m-250 *μ*m. The thickness of the inclined holes was about 1.1 mm-1.3 mm. The aperture was between 50 *μ*m-110 *μ*m, and the inclination angle of inclined holes was between 35° and 80°. The cornified epidermal layer can resist the instant impact from the ground. The oblique hole layer of hoof capsules can store, release, and dissipate the impact energy by deforming itself [28]. They cooperate with each other to realize the excellent buffering and vibration reduction function of the hoof capsules.

Based on the special structure of hoof capsules, a novel bionic cushion for the robot was proposed (Figure 4(a)). The bionic cushion was a hollow cylinder with evenly distributed oblique holes. The angle between the oblique hole and the horizontal direction was *θ* (Figure 4(b)). When the robot was impacted by the ground, the designed cushion with oblique holes could deform in the annular direction, which caused a rotation moment. This rotational torque was transmitted to the sole, so that the sole and the ground rotated relative to each other. At this time, the sliding friction force would consume part of the impact energy. In this process, part of the impact energy was converted into the internal energy of the cushion, and the other part was consumed by friction.

Inspired by the unique biological structure of the hoof capsule, a new bionic vibration damping foot was designed (Figure 5). The bionic foot was composed of the connecting block, bionic cushion, bionic foot sole, steel ball, ball cap, and screw. The bionic foot sole was used to imitate inverted V shape of hoof capsules. Bionic cushion mimicked an oblique hole layer to store energy. In addition, the steel ball, ball cover, and other parts were used to form a similar bearing structure, which ensured that the robot legs would not rotate when the impact energy was consumed by friction. The bionic foot was located at the bottom of the leg robot, which was the part of the robot direct to the ground. It was bolted to the calf of the legged robot. The bionic foot had to withstand the weight of the entire robot and the impact from the ground.

## 3. Simulation Analysis of Bionic Foot

The Abaqus was used to make the finite element simulation analysis. The inclined hole angle (*θ*) of bionic vibration damping feet was set as 30°, 60°, and 90°, respectively. There was no bionic foot sole and cushion with holes in the ordinary foot (Figure 6). An equivalent mass block was added to the upper part of the bionic vibration damping feet, whose mass was equal to the mass of a normal robot. The distance between the bottom of the bionic foot and the ground was set as 1 mm. The robot foot crashed into the ground at 1 m/s to imitate the situation where the robot's foot was impacted by the ground. The coefficient of friction between the robot's feet and the ground was set to 0.1. The material parameters of FEM models in the Abaqus are displayed in Table 1. The soft linear elastic material was used as the material of the bionic cushion to facilitate its ability to absorb impact energy. The material of the bionic sole and the mass block was steel while the material of the ground was rock.

The kinetic energy, frictional dissipation energy, and ground reaction force were selected as indexes to evaluate the buffering effect of the reported bionic foot. The kinetic energy-time curves of the impact process are shown in Figure 7. When the robot feet are not in contact with the ground, there was no change in kinetic energy. After the impact, the kinetic energy began to decline sharply, then increased, and fluctuated steadily. The residual kinetic energy of bionic vibration reduction robot feet was smaller than that of the ordinary one, and the residual kinetic energy decreased with the reduction of angle. This suggested that the proposed bionic structure worked, allowing the bionic foot to consume more kinetic energy than the ordinary foot. The frictional dissipation energy-time curves of bionic vibration reduction feet in the impact process are displayed in Figure 8. The frictional dissipation energy of the bionic vibration damping feet was greater than that of the ordinary one, and they increased with the decrease of inclination. This indicated that the buffering effect of bionic feet increased with the decrease of the angle of inclined holes. As can be seen from Figure 9, the 90° hole structure was not suitable for the buffering and vibration reduction of the bionic foot in the vertical direction. This was consistent with the results of previous studies [27].

The time curves of the ground impact force that an ordinary foot and bionic feet suffer from are shown in Figure 9. The peak impact force of bionic feet was less than that of the ordinary foot, and the peak force decreased with the decrease of the inclination angle. This displayed that the inclination angle was related to the amount of consumed and stored energy of the bionic cushion. When the inclination angle of the bionic cushion was smaller, it was better at absorbing and consuming impact energy. Compared with the ordinary foot, the bionic feet had a longer cushion time, which was beneficial to the stable operation of the robot. All the above results indicated that the proposed bionic feet had good cushion effect.

In order to evaluate vibration reduction performances of the proposed bionic foot, the displacement change of robots after impact and the natural frequency were selected as indexes to make vibration response analysis. The displacement curves of the mass block on the bionic feet and the ordinary foot after impact are displayed in Figure 10. The displacement change of the mass block on the bionic feet was smaller than that of the ordinary one. There was a little difference in the displacement change of the bionic foot with 90° holes and the ordinary one. The bionic foot with 30° inclined holes has the smallest change in displacement. This indicated that the bionic foot could better reduce the vibration caused by ground impact. The first ten-order natural frequencies of the bionic feet and ordinary foot were obtained through modal analysis (Figure 11). It could be seen from Figure 11 that the first three-order natural frequency of bionic feet was smaller than those of the ordinary foot, and the natural frequency gradually decreased with the decrease of the angle of inclined holes.

The parameters of the first ten-order vibration model for a normal foot and bionic feet are displayed in Tables 2–5. After being impacted, the first-order and second-order vibration modes of the robot foot were mainly translational movements of *X* and *Z*. In other words, the first-order and second-order vibration of the ordinary foot and bionic feet was mainly translational motion in the *x*‐*z* plane. For buffering and vibration reduction feet with 30° and 60° inclined holes, the translational motion in the *Y* direction played a leading role in the third-order and fourth-order modes. For the ordinary foot and bionic foot with 90° inclined holes, the main vibration mode of the third order was the rotation in the *Y* direction. Their fourth-order vibration mode was similar to that of the bionic feet with 30° and 60° inclined holes. The vibration in the translational direction of *Y* played an important role. The vibration mode after the fourth order was complex and changeable where the vibration participation coefficient was small, so its vibration influence can be ignored.

Compared with the normal foot, bionic vibration reduction feet with inclined holes had smaller first three natural frequencies, which help it to obtain a larger damping range. According to the parameters of vibration mode, the structure of the inclined hole changed the main vibration form of the third order. The bionic structure transformed the main vibration mode of the third order from rotation in the *Y* direction into translational motion. This may be because the structure reduced the stiffness of the bionic foot in the *Y* direction. In summary, the inclined hole feature changed the natural frequency of the bionic foot, expanded the frequency range of vibration reduction, and facilitated the absorption of vibration energy.

## 4. Conclusions

The microstructure of goats' hoof capsules was carefully observed. The unique shape of hoof capsules increased the contact area with the ground and friction, which was better to reduce impact power. The internal oblique hole features enabled the hoof capsules to absorb energy through appropriate changes after impact. Based on the above research, a bionic foot for buffering and vibration reduction of legged robots was proposed. Compared with the ordinary foot, bionic feet could better use elastic deformation and the friction force to consume the impact energy, which was better for the walking stability of legged robots. In addition, the bionic foot effectively reduced the vibration of the robot caused by impact. The natural frequency of the bionic foot was smaller than that of the ordinary foot, which ensured that the bionic foot has a wider range of vibration reduction.

## Figures and Tables

**Figure 1:** The picture of the goats' hoof capsules: the bottom (a) and the top (b).

**Figure 2:** The design and bionic prototype of foot sole:(a) the touchdown contour of nails and (b) the bionic foot sole.

**Figure 3:** SEM pictures: the hoof capsules (a), the inclined holes in the hoof capsules (b), the diameter of the inclined holes (c), and the bottom of hoof capsules (d).

**Figure 4:** The schematic diagram: the bionic cushion (a) and the angle of oblique holes (b).

**Figure 5:** The bionic foot: the unassembled model (a) and the assembled model (b).

**Figure 6:** Ordinary robot foot.

**Figure 7:** Kinetic energy-time curves of different robot feet.

**Figure 8:** Time curves of frictional dissipation energy of different robot feet.

**Figure 9:** Time curves of ground impact force of different robot feet.

**Figure 10:** The displacement curves of the mass block on the bionic feet and the ordinary foot after impact.

**Figure 11:** Natural frequencies of the bionic feet and ordinary foot varying with orders.

**Table 1:** Material parameters of bionic cushion, bionic foot sole, ground, and mass block.

Model	Modulus of elasticity (MPa)	Poisson's ratio	Density (kg/m^3^)
Bionic cushion	7.84	0.47	1200
Foot sole	2.1 × 10^5^	0.3	7800
The ground	4 × 10^4^	0.25	2500
Mass block	2.1 × 10^5^	0.3	50000

**Table 2:** Participation coefficients of all vibration modes of the ordinary foot.

Mode	*X*	*Y*	*Z*	*X*‐*R*	*Y*‐*R*	*Z*‐*R*
1	0.57566	−8.06*E* − 09	0.65584	−2.29*E* − 03	2.18*E* − 02	2.01*E* − 03
2	0.65584	1.95*E* − 08	-0.57566	2.01*E* − 03	1.60*E* − 03	2.29*E* − 03
3	2.02*E* − 09	−2.36*E* − 06	−1.84*E* − 08	4.20*E* − 08	1.16*E* − 02	4.13*E* − 08
4	4.92*E* − 08	1.00*E* − 05	1.93*E* − 09	−1.79*E* − 07	7.48*E* − 10	−1.76*E* − 07
5	−6.19*E* − 07	−1.52*E* − 07	−7.35*E* − 07	−2.30*E* − 09	−2.39*E* − 08	4.88*E* − 09
6	6.96*E* − 07	1.56*E* − 07	−6.66*E* − 07	−5.05*E* − 09	6.87*E* − 10	−7.83*E* − 09
7	−3.01*E* − 06	−1.61*E* − 07	−3.07*E* − 06	−4.48*E* − 08	−1.07*E* − 07	5.06*E* − 08
8	−3.04*E* − 06	−1.45*E* − 07	3.04*E* − 06	5.08*E* − 08	−1.08*E* − 09	4.98*E* − 08
9	8.59*E* − 07	8.22*E* − 09	8.66*E* − 07	1.06*E* − 08	3.05*E* − 08	−1.03*E* − 08
10	8.64*E* − 07	7.10*E* − 09	−8.63*E* − 07	−1.03*E* − 08	2.62*E* − 10	−1.09*E* − 08

**Table 3:** Participation coefficients of all vibration modes of the bionic foot with 90° inclined holes.

Mode	*X*	*Y*	*Z*	*X*‐*R*	*Y*‐*R*	*Z*‐*R*
1	-0.53999	8.71*E* − 07	0.75897	−2.65*E* − 03	3.68*E* − 03	−1.88*E* − 03
2	0.75896	−1.63*E* − 07	0.53999	−1.88*E* − 03	2.30*E* − 02	2.65*E* − 03
3	−2.52*E* − 06	−2.73*E* − 03	3.25*E* − 06	4.87*E* − 05	1.13*E* − 02	4.79*E* − 05
4	−3.39*E* − 06	1.122	−8.44*E* − 07	−2.00*E* − 02	1.81*E* − 05	−1.97*E* − 02
5	−2.01*E* − 06	−1.69*E* − 02	2.03*E* − 06	3.01*E* − 04	−3.38*E* − 06	2.96*E* − 04
6	4.92*E* − 03	−8.08*E* − 07	−7.04*E* − 03	−1.95*E* − 04	−3.56*E* − 05	−1.14*E* − 04
7	−7.03*E* − 03	9.64*E* − 06	−4.93*E* − 03	−1.14*E* − 04	−2.12*E* − 04	1.95*E* − 04
8	−1.07*E* − 06	−5.36*E* − 06	1.81*E* − 06	1.50*E* − 07	1.49*E* − 08	1.27*E* − 07
9	−1.49*E* − 06	3.41*E* − 03	9.02*E* − 07	−6.07*E* − 05	3.82*E* − 06	−5.97*E* − 05
10	1.85*E* − 03	5.20*E* − 07	2.49*E* − 03	7.73*E* − 05	7.65*E* − 05	−6.28*E* − 05

**Table 4:** Participation coefficients of all vibration modes of the bionic foot with 60° inclined holes.

Mode	*X*	*Y*	*Z*	*X*‐*R*	*Y*‐*R*	*Z*‐*R*
1	0.99313	1.69*E* − 05	0.38694	−9.03*E* − 04	2.45*E* − 02	3.81*E* − 03
2	-0.38693	−2.33*E* − 05	0.99313	−3.81*E* − 03	1.05*E* − 02	−9.03*E* − 04
3	6.34*E* − 05	-0.19575	−2.51*E* − 05	3.49*E* − 03	1.09*E* − 02	3.43*E* − 03
4	4.37*E* − 05	1.1251	8.29*E* − 05	−2.01*E* − 02	1.49*E* − 03	−1.97*E* − 02
5	-0.31171	−2.83*E* − 05	0.36829	9.73*E* − 03	8.98*E* − 04	3.19*E* − 03
6	0.36827	−5.76*E* − 04	0.31159	3.20*E* − 03	1.20*E* − 02	−9.71*E* − 03
7	1.39*E* − 04	9.18*E* − 02	7.17*E* − 04	−1.62*E* − 03	1.82*E* − 04	−1.62*E* − 03
8	−7.79*E* − 02	1.12*E* − 03	1.93*E* − 02	9.91*E* − 04	−1.05*E* − 03	1.32*E* − 03
9	−2.04*E* − 02	1.33*E* − 03	−7.79*E* − 02	−1.36*E* − 03	−1.73*E* − 03	1.01*E* − 03
10	−4.37*E* − 04	−9.85*E* − 04	1.38*E* − 03	4.80*E* − 05	1.48*E* − 05	1.40*E* − 05

**Table 5:** Participation coefficients of all vibration modes of the bionic foot with 30° inclined holes.

Mode	*X*	*Y*	*Z*	*X*‐*R*	*Y*‐*R*	*Z*‐*R*
1	0.74848	1.09*E* − 05	0.53125	−1.69*E* − 03	2.27*E* − 02	3.48*E* − 03
2	-0.53126	−1.00*E* − 05	0.74849	−3.48*E* − 03	3.65*E* − 03	−1.69*E* − 03
3	4.60*E* − 06	-0.27758	5.75*E* − 06	4.95*E* − 03	1.03*E* − 02	4.87*E* − 03
4	−5.27*E* − 05	1.0762	−4.47*E* − 06	−1.92*E* − 02	2.10*E* − 03	−1.89*E* − 02
5	0.47678	1.66*E* − 04	0.17528	−1.16*E* − 03	1.16*E* − 02	−9.12*E* − 03
6	0.17526	1.42*E* − 05	-0.47668	−9.12*E* − 03	−5.23*E* − 03	1.16*E* − 03
7	−3.48*E* − 05	5.77*E* − 05	−5.28*E* − 05	−1.43*E* − 06	−1.35*E* − 06	−9.43*E* − 08
8	−3.96*E* − 02	3.18*E* − 04	−8.42*E* − 02	−8.59*E* − 04	−2.18*E* − 03	9.57*E* − 04
9	8.41*E* − 02	4.06*E* − 05	−3.95*E* − 02	−9.62*E* − 04	8.07*E* − 04	−8.53*E* − 04
10	3.63*E* − 05	7.08*E* − 02	1.78*E* − 04	−1.26*E* − 03	3.27*E* − 04	−1.24*E* − 03

## Data Availability

The data used to support the findings of this study are available from the corresponding author upon request.
